RETRACTED

# Assessing the Influencing Factors of Electronic Word-of-Mouth on CSR Issues. A Case of Hospotality Service Industry of China

**DOI:** 10.3389/fpsyg.2022.924779

**Published:** 2022-06-21

**Authors:** Zhuo Liu, Suihuai Yu, Fangmin Cheng, Rida Waheed

**Affiliations:** ^1^School of Art and Design, Tianjin University of Technology, Tianjin, China; ^2^School of Mechanical Engineering, Northwestern Polytechnical University, Xi’an, China; ^3^Department of Finance and Economics, College of Business, University of Jeddah, Jeddah, Saudi Arabia

**Keywords:** CSR, eWOM, social networking sites, structural model, Wechat, China

## Abstract

Corporate social responsibility (CSR) information can be effectively disseminated via social media in a variety of industries, including the hospitality sector. In the same way, the media has a significant impact on CSR because the news media helps companies achieve their CSR goals. Prior research has not examined the main factors that influence electronic word of mouth (eWOM) on media coverage of CSR issues via social networking websites. For the purpose of examining the most significant predictors of intention to share or comment on negative CSR news reported by one media outlet on a specific social networking site (SNS). 677 Wechat users in China were surveyed in order to test the proposed model empirically. According to the findings of the study, eWOM intentions are positively influenced by environmental CSR content, and advertisement related CSR content. It also confirmed that the value of information is positively influenced by the credibility of the source. The variables interpersonal influencer impact and privacy concerns had no significant relationship, nor did they have any significant relationship with the intentions to share and comment on Wechat. Further the study findings suggest the theoretical and managerial policy recommendation for decision makers.

## Introduction

Social media has developed as a powerful and effective instrument for disclosing information about a company’s social responsibility (Wu and Zhu, 2021). Additionally, Newspapers and periodicals, for example, have set up their pages on social media sites like Facebook, Instagram, Wechat to interact with their target readers (Fatma et al., 2020), making CSR information readily available (Wang et al., 2022). People worldwide are using social media to share information on corporate social responsibility. People can use this media to develop content or openly express their thoughts on CSR-related topics as a result of this freedom (Camilleri, 2021). In order to better engage customers and other stakeholders, companies can use CSR engagement as a unique communication strategy to build positive associations between their corporate and product brands (Bellini et al., 2020; Huang et al., 2021; Castro et al., 2022). However, companies increasingly use social media to advertise their CSR commitment (Castillo-manzano et al., 2021).

RETRACTED

We shouldn’t be surprised that businesses have begun utilizing social media marketing strategies in response to the explosive growth of social media adoption. These include marketing strategies such as public relations and advertising in addition to community engagement and corporate social responsibility (Camilleri, 2022). More support for a CSR program could be gained by including customers in communicating about it (Aktan et al., 2022). eWOM on CSR information has been given a new dimension by SNSs, which enable users to share with their existing networks before, during, and after travel (Yusuf et al., 2018).

Customer feedback has never been more accessible to businesses than it is now, thanks to the power of social media. Customer reviews can be posted on e-commerce websites, social media platforms, weblogs, and peer-to-peer networking sites. Electronic word-of-mouth is enriched by client feedback and opinions about a product or service. There are various ways to disseminate eWOM, including likes, comments, ratings, reviews, videos, tweets, photos, and blog articles. In the eyes of Internet users, eWOM is more trustworthy than traditional media (Khan, 2018). Online reviews play a significant role in determining a customer’s ultimate purchase decision (Weihong et al., 2021). eWOM characteristics must be addressed for a company’s expansion to be successful. To Hootsuite’s Global State of Digital 2019 Report (2019), there were 3.484 billion social media users wide-reaching, with an annual growth rate of 9%. Despite an increasing interest in social media studies. It’s still not obvious how customers’ CSR-related social media activities inspire their approaches and behaviors toward products (Ali et al., 2019; Murtafi’ah and Putro, 2019; Deng and Zhao, 2022). Consumers’ CSR-related behaviors on social media are examined in this study to see if they affect their intention, brand attitude, and purchase intention.

In this way, this research focuses on hotel CSR communication over the Internet, an area that is increasingly being studied but is still considered under-researched. For the sake of this investigation, we concentrate on the elements that influence the intention to develop eWOM on CSR concerns (a firm’s post on environmental CSR) covered by hotel firms via a specific SNS (social network). The Stimulus-Organism-Response (S-O-R) model is the foundation for the suggested model (Bolaños et al., 2022). We are interested in how Wechat users and the content’s characteristics influence their responses (intention to share). According to this study’s explanatory variables, information processing is influenced by users’ attitudes toward sharing both commercial and environmental CSR information, homophily, and expressive information sharing (Chen et al., 2018).

RETRACTED

Rest of the study is organized as follows: The conceptual model and the hypotheses tested are discussed in the section “Literature and Research Hypotheses”. In section “Methodology,” the authors will detail the sample features and the process of data assembling, and the measured variables. Section “Results and Discussion” provides the findings of the study. Finally section “Conclusion and Policy Implications” discuss the theoretical and managerial implications.

## Literature and Research Hypotheses

Corporate social responsibility is based on a more beneficial impact on society and a greater awareness of the social and ethical ramifications of a company’s activities (Sendlhofer, 2020). There are four key obligations in Carroll (1996) “s model of” corporate social responsibility (CSR). These are the pursuit of profit, compliance with legal and ethical requirements, and charitable giving. According to Wu and Zhu (2021), three of the most popular kinds of CSR include charitable donations, improved workplace standards, and environmental activities. Based on the work of Schramm-Klein et al. (2015), this study examines aspects of corporate social responsibility (CSR) that may be more apparent in social media contexts.

In recent years, new media technologies like the Internet have made it easier for consumers to interact with friends and acquaintances from their existing social networks and meet new people online (Bocquet et al., 2019). eWOM, or electronic word-of-mouth, has taken off as a result of the rapid growth of the Internet. This includes all informal conversations with consumers via Internet-based technologies related to the use or quality of specific goods and services, or their sellers, as described by Dalla-Pria and Rodríguez-de-Dios (2022). Consumers’ interactions with one another and with manufacturers are included in this definition, too. In the eyes of many, electronic word-of-mouth (eWOM) is a trustworthy resource. Consumers’ expectations, preferences, and attitudes are said to be influenced by eWOM, which, in turn, impacts the purchasing and post-use evaluation judgments (Hui, 2008). A wide range of eWOM examples includes emotional support, empathy, generosity, a sense of belonging, and self-esteem, which entails the engagement of actors whose behavior is motivated by various factors (Castka et al., 2004). We have very little theoretical understanding of eWOM in CSR communication via social media (e.g., SNS) despite earlier studies in the hospitality industry providing insights into the motivations and effects of eWOM behavior (Carlini et al., 2021).

RETRACTED

In order to contribute to a more sustainable future, companies should consider the priorities of CSR (Anser et al., 2018). It is possible to categorize the marketing outcomes of CSR communication into two distinct groups: those related to the brand and corporate mentality and those related to the viral transmission of the message, which is essential to a successful social media campaign. Communication about corporate social responsibility (CSR) has been beneficial to impact how customers feel about a company’s branding and products (Crowther et al., 2018). Consumers see socially responsible companies positively (Rajesh, 2020; Khan et al., 2021). Brand and product attitudes and behavioral intentions are influenced positively by CSR advertising, promoting a good image of the organization (Wang and Sarkis, 2017; Elshabasy, 2018).

Researchers have analyzed and categorized different social media content (Úbeda-García et al., 2021), CSR sharing and participation are still low. However, CSR issues like the environment and education are more commonly discussed on social media (Yusliza et al., 2019). This is even though CSR sharing and engagement are still low (Castro et al., 2022). EWOM has been demonstrated to increase the virality of a CSR post by sharing or endorsing it because of its favorable impact on believability (Yumei et al., 2021). As a result, the legitimacy of CSR, its motivations, and the corporate and brand attitudes that go along with them will be enhanced, as will social media support through likes, comments, and shares.

This research investigates how the response is influenced by elements linked to the recipients (Wechat users) and the stimuli (post content) (intention to share).

### Social and Environmental Awareness

According to this survey, CSR is defined as how customers engage in CSR communication via social media from companies. Consumer friends may like or follow the CSR activities on social media, write or share comments about a company’s CSR activities, or join groups dedicated to a brand’s CSR activities, for example. Consumer involvement and viral advertising have been found to benefit from the use of social media (Stanislavská et al., 2020). CSR efforts and customer interaction can be promoted through social media fan sites created by firms such as McDonald’s, Starbucks, and Nike. Consider the Clean Water Project, an initiative by Coca-Cola to address the issue of unsafe drinking water for rural children by establishing a corporate Facebook page. They are more inclined to be loyal to a firm if they follow, like, or sign up for these social media accounts and follow them and are more open to receiving information about it. Consumers can also help spread word of mouth about a brand’s CSR efforts by forwarding other people’s comments on the topic.

eWOM comments on Wechat about negative corporate social responsibility (CSR) material, such as allegations of environmentally harmful activity, have been the subject of several studies. When it came to attitudes regarding posting comments on CSR on Facebook, (Mohamud, 2018), for example, discovered that environmental awareness and social awareness had a direct and beneficial impact on attitudes but not on how valuable people perceived that data to be.

RETRACTED

According to key research (Bagh et al., 2017) we’ve used the findings to increase customer knowledge of corporate social responsibility (CSR). There is substantial evidence that CSR dimensions are linked to good e-WOM.

**H1:** Consumers CSR related activities are positively influenced by social awareness.

**H2:** Advertisement-related content on SNSs is highly influenced by social awareness.

**H3:** Environmental CSR content is highly influenced by environmental awareness.

**H4:** Advertisement-related content on SNSs is highly influenced by environmental awareness.

### Information Sharing

Internet-based word of mouth (WOM) interaction is known as eWOM, or electronic word of mouth (Kong et al., 2020). Consumers spread service information and product directly and indirectly while using eWOM, similar to offline WOM. eWOM, on the other hand, makes use of the Internet as a middleman to expedite the dissemination of information compared to more traditional word-of-mouth approaches (Yusuf et al., 2018). Six social relationship elements have been identified in earlier studies as motivating eWOM behavior: tie-strength, compliance, social capital, and trust (Aktan et al., 2022).

Tie-strength describes the degree to which network members are intimately connected, as measured by eventually spent together, the passion of feelings experienced by each member, and the degree of intimacy experienced by the network as a whole.

Conformity is people’s propensity to emulate the conduct of a group, even if the group’s principles and practices do not match their attitudes and ideas, which is known as groupthink.

Social capital, On SNSs, long-term, organized individual interactions in a social network provide people with the resources they need (Irfan et al., 2022). Bridging and bonding are two types of social capital (Iqbal et al., 2021). Social capital is produced through reciprocal data interchange across groups of people from different backgrounds, which is why it is called “bridging social capital” (Hou Yumei et al., 2021). Bonding social capital, on the other hand, social standards and emotional support among members of a homogeneous group are highlighted (Iqbal et al., 2020).

RETRACTED

Trust it’s characterized as “a willingness to place trust in a trading partner” (Khoso et al., 2021). eWOM information is analyzed by SNS users depending on the trustworthiness of the data source while exchanging service and product data on SNSs (Huang et al., 2022). As a result, people’s trust in their SNS friends significantly impacts their eWOM activity on SNSs.

**H5:** EWOM behavior is influenced by SNS users’ ties to their SNS buddies.

**H6:** eWOM conduct will be positively influenced by SNS users’ agreement with their SNS peers.

**H7:** eWOM behavior of SNS users will be influenced favorably if SNS users intend to (a) channel and (b) link their social capitals on SNSs.

**H8:** EWOM behavior is influenced by SNS users’ trust.

### Interpersonal Influence

The influence of SNS friends on individuals is an essential topic in eWOM literature (Tang et al., 2022). Interpersonal impact comes in normative and informative flavors (Graafland and Smid, 2014). The predisposition to accept the dynamic norms and expectations is normative influence. In contrast, the degree to which one acquires service and product information from competent individuals is called informational influence (also known as informational learning) (Zhang et al., 2015; Abubakar et al., 2022). EWOM communications impacted by SNS friends’ norms and values influence customers who are sensitive to normative impacts. Consumers are more likely to rely on eWOM information from SNS friends who know about the topic (Chaudhary and Akhouri, 2018; Lu et al., 2021).

**H9:** User eWOM behavior will be positively influenced by (a) normative and (b) informative influences on SNS users.

### Attitudes Toward CSR Communications

People’s perceptions and opinions about online information were examined by researchers using the Theory of Reasoned Action and the related Theory of Planned Behavior (Liao et al., 2018; Zhuang et al., 2021). A person’s attitude is the degree to which they have a favorable or unfavorable view of the prospective outcomes of specific activities (Mattera et al., 2020). According to this line of reasoning, people may be prone to having biased judgments because they are aware of and informed about various subjects (Kemper et al., 2013). Li et al. (2020) argued in a similar vein that people’s attitudes frequently come before their evaluations.

RETRACTED

Corporate social responsibility (CSR) communications elevate society’s expectations and put firms under heightened obligation to demonstrate their legitimacy and social license to operate (Chahine et al., 2021). If stakeholders do not believe in a company’s CSR credentials, the two can have a negative relationship (Meseguer-Sánchez et al., 2021). Communications on corporate social responsibility can be seen as either positive or negative depending on stakeholders’ perceptions (Collier and Esteban, 2007; Agyemang and Ansong, 2017; Le, 2022; respectively).

**H10:** People’s opinions regarding online CSR communications are influenced by the relevance of their presented material.

### Impact of Influencers

The influencer’s popularity may be influenced by factors other than the number of people who follow them. According to popular literature, there are some “rules” regarding who to follow and how many followers you should have compared to how many followers you should have on Twitter. You should follow persons with a favorable follower-to-follower ratio or those who have more followers than the accounts they follow. However, following several accounts provides the user with a greater opportunity to learn about various issues and viewpoints, which may be advantageous in terms of opinion leadership (Graafland and Smid, 2014). However, following too many individuals isn’t a good idea because it’s unlikely that you’ll be able to keep up with all of their updates.

**H11:** We expect an influencer with a large number of followers to have a favorable impact on the likeability of the influencer.

## Methodology

### Questionnaire Development

The data for the study is gathered through a conventional survey questionnaire. Women and men of all ages and educational levels are included in the demographic portion of the table. Both emotional commitment and positive e-WOM are measured in the second half of the survey. Likert scale responses ranged from “strongly disagree” to “strongly agree” on a seven-point scale. Based on their input and recommendations, hospitality administration students reviewed the initial questionnaire to ensure its content validity (see Appendix A1).

Valid and reliable methods from the literature have been adapted to measure the study’s constructs: CSR dimensions from Osei-Kojo and Andrews (2020); affective commitment from Martínez-Ferrero et al. (2015), Tiep Le et al. (2021), and positive eWOM from Fifka and Pobizhan (2014), Kang et al. (2021). Each and every one of the structures reflect the underlying idea. It was decided to gauge the worth of data by using three elements from Utami and Hasan (2021) as a starting point. A scale based on studies by Hong et al. (2016) was used to measure attitudes toward sharing and commenting. Wechat users make up the survey universe; therefore, we referenced the 2017 Annual Study of Social Networks to ensure the most accurate facts. CSR-related social media activities, consumer identification with the brand, brand attitude, eWOM intention, and purchase intention were all examined in an online survey of general Chinese consumers.

RETRACTED

### Respondents’ Selection and Sample Size

Only Chinese social media users were polled for this study on CSR and social media. 631 legitimate responses were received from 722 qualified Chinese social media users in the online survey. The samples were taken in December of last year. At 631 people, around 55% of those polled agreed to participate in the survey, with the remaining 45% disagreeing. The respondents’ ages ranged from 19 to 65 years old, with a mean of 31 years older. Convenience sampling was used for one pre-test (university students). Wechat users were explicitly targeted in this study, and 25 university students were recruited to help determine whether the stimulus was realistic and provide feedback on the questionnaire. Wechat users were asked to reply to a survey after being presented an incentive in the form of a false article from a newspaper. In China, Tencent has developed the WeChat social media app as well as an instant messaging and mobile payment service. It was first introduced in 2011 and has since grown to become the world’s largest standalone mobile application in 2018, with more than 1 billion monthly active users worldwide.

### Statistical Analysis

Smart PLS (v.3.2.7) and IBM SPSS were used to analyze the data (v.24.0). SEM’s second-generation PLS technique, also known as a variance-based approach, is more robust and advanced than its first-generation SEM counterpart (Haghighi and Pour, 2014). PLS-SEM is a good option for this investigation because of its capacity to deal with intricate structural models. PLS-SEM was also chosen to owe to its capacity to instantaneously examine all the causal links of the underlying components while simultaneously addressing measurement errors (Garcia et al., 2017; Zhang et al., 2019). It is also important to note that this research’s purpose is exploratory; hence PLS-SEM is an appropriate choice (Agudo Valiente et al., 2012). For this investigation, following (Agudo Valiente et al., 2012) guidelines for PLS-SEM best practices, all measurement models were examined separately before the primary structural model was considered. Additional tests will be conducted (e.g., data screening for missing values and out-liars, common-method variance test and non-response bias test, etc.) to assure the quality of the data, alongside additional verifications of trustworthiness and accuracy. Data screening and pre-analytics in this study continue to be discussed.

RETRACTED

### Non-response Bias Test

This study used a self-administered survey-based questionnaire for data collection, as described in the previous section. 65.5 percent of those who responded to our survey did so. As a result, it is critical to analyze whether the data used in this study have any non-response bias. Excessive non-response bias can be checked by using the extrapolation method. In cross-sectional research, Armstrong and Overton (1977) employ the extrapolation approach to determine non-response bias. This method entails comparing the mean values of early and late participants in a study to determine if any variation in the mean values of any of the components concerned. IBM SPSS was used to execute a separate *t*-test to compare the means of our first 100 respondents with our last 100 respondents (v.24.0). According to the findings, both sub-groups’ mean values did not differ significantly (p 0.05). This study does not suffer from non-response bias, according to these findings.

### Common-Method Variance Test

Cross-sectional studies face a severe problem with common-method variance (Hens et al., 2018). Dey et al. (2018) guidelines were used to check for any common-way modification in this research, thus addressing this issue. As a single factor analysis, we applied IBM SPSS’s varimax alternation approach to conducting Harman’s (1976) one-factor test on each of our 32 components (v.24.0) scale. Five components emerged from the dataset: CSR, employee engagement, organizational pride, organizational identity, and DSIW. The rotation converged in seven iterations. This study’s findings show that common-method variation is not an issue.

## Results and Discussion

### Descriptive Analysis, Correlation Analysis

A gender-balanced sample of 640 responses showed a male preponderance of 56% and a female preponderance of 44%. The majority of our respondents (nearly 39 percent) were between 31 and 35. Only 8% of our respondents had less than 5 years of work experience, based on overall work experience data. More than half of our respondents were in non-management roles, followed by 20% first-line managers and 9% middle-level managers. As for the respondents’ formal educational qualifications, we discovered that 39 percent had bachelor’s degrees, 23 percent had graduate degrees, and 24 percent had only completed high school. In addition, our sample consisted of 48 percent Malaysians, 26 percent Indians, and 24 percent Chinese, which demonstrates a great blend of the three major Asian nationalities that call Malaysia home. Table 1 also contains comprehensive data on the demographic characteristics of our survey participants.

RETRACTED

**TABLE 1:** Demographic attributes.

Variables	Category/Distribution	Frequency	%
Gender	Male	402	59%
	Female	275	41%
	Total	677	100%
Age	> 24	42	6%
	25–30	156	23%
	31–35	261	39%
	36–40	165	24%
	< 40	53	8%
	Total	677	100%
Work Experience	> 5	63	9%
	10-May	184	27%
	11–15	242	36%
	16–20	141	21%
	< 20	47	7%
	Total	677	100%
Education level	Bachelor’s degree	161	24%
	Diploma	275	41%
	High School	158	23%
	Master’s degree	59	9%
	Others	24	4%
	Total	677	100%
Job title	Senior Manager	29	4%
	Middle Manager	62	9%
	First-line Manager	139	21%
	Non-Managerial Employee	345	51%
	Others	102	15%
	Total	677	100%

### Reliability Analysis

(Agudo Valiente et al., 2012) developed a method for determining discriminant validity that compared the variance retrieved for each set of components with the squared association approximation between the two concepts (AVE coefficient). As a result, the scales used to assess each idea were discriminatively valid, as the variances obtained were always larger than the squared correlation between the concepts. For both the Bentler–Bonett normed and non-normed models, the factorial model’s fit indexes exceeded the minimum value of 0.9. It was also deemed acceptable that the RMSEA and normed complied with the requirements. Scale reliability was assessed using Cronbach’s alpha, compound reliability, and AVE coefficients. Silvestri and Veltri (2020) observed that all of these statistics were over the required minimum of 0.7 and 0.5, proving the constructs’ internal reliability. All of the scales had standardized lambda coefficients greater than 0.5 and were deemed statistically significant at a 95% confidence level. Table 2 displays the latent constructs’ reliability, validity, and relationships in detail. Table 3 additionally includes correlations between all detected variables (i.e., indicator correlations matrix).

**TABLE 2:** Reliability and validity.

Latent construct(s)	Cronbach’s alpha	CR	AVE
Impact of influencers	0.863	0.894	0.514
Social awareness	0.72	0.827	0.545
Environmental Awareness	0.871	0.896	0.561
Information Sharing	0.801	0.858	0.503
Attitude	0.71	0.838	0.633

**TABLE 3:** Correlations among latent constructs.

Latent constructs	Impact of influencers	Social awareness	Environmental awareness	Information sharing	Attitudes
Impact of influencers	1				
Social awareness	0.796	1			
Environmental Awareness	0.866	0.81	1		
Information Sharing	0.836	0.78	0.843	1	
Attitude	0.784	0.709	0.764	0.759	1

A approach established by Fornell and Larcker (1981) was used to assess the discriminant validity of the scales. This procedure demands a comparison of the variance extracted for each pair of constructs (AVE coefficient) with the squared correlation estimate between these two constructs (Table 4). It was found in all cases that the variances recovered for each concept were bigger than the squared correlation between them, indicating that the measurement scales had discriminant validity (see Table 5)

RETRACTED

**TABLE 4:** Correlations among observed variables/indicator correlations matrix.

	IMI 1	IMI 2	IMI 3	SOAW 1	SOAW 2	SOAW 3	ENA 1	ENA 2	ENA 3	ENA 4	INSA 1	INSA 2	INSA 3	INSA 4	ATU 1	ATU 2	ATU 3
IMI 1	1																
IMI 2	0.534	1															
IMI 3	0.514	0.417	1														
SOAW 1	0.49	0.437	0.37	1													
SOAW 2	0.512	0.391	0.447	0.371	1												
SOAW 3	0.456	0.402	0.308	0.326	0.379	1											
ENA 1	0.545	0.498	0.45	0.392	0.472	0.361	1										
ENA 2	0.542	0.538	0.476	0.412	0.442	0.378	0.491	1									
ENA 3	0.499	0.428	0.421	0.399	0.369	0.354	0.408	0.418	1								
ENA 4	0.421	0.412	0.349	0.343	0.337	0.359	0.383	0.414	0.309	1							
INSA 1	0.507	0.444	0.429	0.394	0.384	0.347	0.455	0.451	0.378	0.34	1						
INSA 2	0.543	0.488	0.433	0.399	0.419	0.377	0.502	0.49	0.419	0.429	0.471	1					
INSA 3	0.467	0.421	0.364	0.309	0.363	0.348	0.442	0.374	0.325	0.283	0.375	0.417	1				
INSA 4	0.501	0.422	0.403	0.395	0.369	0.351	0.435	0.393	0.38	0.369	0.391	0.475	0.364	1			
ATU 1	0.466	0.422	0.417	0.38	0.358	0.324	0.412	0.4	0.37	0.38	0.413	0.411	0.293	0.42	1		
ATU 2	0.504	0.445	0.43	0.394	0.37	0.347	0.487	0.489	0.409	0.401	0.426	0.465	0.376	0.437	0.415	1	
ATU 3	0.597	0.532	0.479	0.486	0.455	0.403	0.52	0.502	0.455	0.414	0.507	0.517	0.409	0.46	0.452	0.511	1

**TABLE 5:** Results of discriminant validity analysis.

	Impact of influencers	Social awareness	Environmental awareness	Information sharing	Attitude
Impact of influencers	0.87				
Social awareness	0.35	0.86			
Environmental awareness	0.13	0.12	0.92		
Information sharing	0.21	0.19	0.11	0.67	
Attitude	0.1	0.09	0.12	0.09	0.85

Additionally, we investigated the cross-loading values of our constructs to verify their discriminant validity. Each measurement item should share its highest loading with its latent construct, rather than the cross-loadings shared with other concepts included in the proposed conceptual model. Cross-loading values for each of our measurement models are listed in Table 6. As advised by Cabral and Sasidharan (2021), all cross-loading values are over the 0.50 criterion (2017). This meets discriminant validity. All of the study’s measurement models were valid and reliable, and this study’s findings meet those criteria. Now, the focus shifts to the evaluation of the structural model used in this research.

RETRACTED

**TABLE 6:** Cross loading values.

	Impact of influencers	Social awareness	Environmental awareness	Information sharing	Attitudes to share content
IMI 1	**0.815**	0.67	0.733	0.714	0.655
IMI 2	**0.744**	0.601	0.651	0.623	0.61
IMI 3	**0.696**	0.555	0.613	0.575	0.533
SOAW 1	0.577	**0.713**	0.59	0.56	0.526
SOAW 2	0.527	**0.681**	0.533	0.506	0.454
SOAW 3	0.598	**0.748**	0.605	0.593	0.52
ENA 1	0.542	0.478	**0.607**	0.522	0.476
ENA 2	0.573	0.549	**0.679**	0.564	0.504
ENA 3	0.557	0.533	**0.643**	0.534	0.498
ENA 4	0.609	0.577	**0.708**	0.581	0.53
INSA 1	0.562	0.498	0.533	**0.649**	0.511
INSA 2	0.573	0.547	0.577	**0.688**	0.536
INSA 3	0.523	0.471	0.547	**0.651**	0.459
INSA 4	0.642	0.621	0.652	**0.753**	0.554
ATU 1	0.624	0.562	0.621	0.609	**0.79**
ATU 2	0.656	0.588	0.628	0.622	**0.815**
ATU 3	0.59	0.542	0.572	0.58	**0.781**

*Bold values indicate the cross loading values.*

### Estimation of Hypothesized Structural Model

Sharing and commenting on CSR-related postings aren’t much impacted by privacy concerns. Since previous research revealed a direct correlation between trust and behavioral intentions in numerous scenarios (Cabral and Sasidharan, 2021). The current research model was developed following Hair et al. (2010) recommendations and included the direct influence of Wechat trust on CSR-related posts being shared or commented on, eliminating the linkages between privacy concerns. According to empirical data, Wechat posts about corporate social responsibility (CSR) are more likely to be shared and commented on if people are more likely to be open about their own experiences. The findings shows that all variable has positive effect on the attitude or intention to share and comment on CSR posts on Wechat moments, according to a preliminary estimation of the structural model. Wechat’s trust does not have an impact on privacy concerns (hypothesis H2). In the proposed research model interpersonal influence has no impact on environmental CSR contents, so this variable has no effect. But the results of the LM Test show that environmental CSR content has a significant and positive impact on people’s intentions to share and comment on content related to CSR, which was not previously hypothesized. Although this relationship is theoretically plausible, previous research has found that trust and behavioral intentions are directly linked in a variety of contexts (Mouzas et al., 2007; Wilkins et al., 2009).

Using the proposed research model as a basis, Figure 1 and Table 7 summarizes the results for the estimation of the structural model, including goodness-of-fit indices for the structural model, R2 statistics for each dependent variable, and the standardized coefficients and significance level (p-value) for each relationship. As a result, the goodness-of-fit indices support the correct definition of the structural model (Normed 2 = 2.32; BBNFI = 0.92; BBNNFI = 0.95; CFI = 0.91; IFI = 0.91; RMSEA = 0.09), explaining a significant proportion of the variance in the dependent variable (BBNFI = 0.92; BBNNFI = 0.95; RMSEA = 0.09). (R2 over 0.50 for intention to share and comment on Wechat posts about CSR).

RETRACTED

**FIGURE 1:** Structural path analysis. Goodness of Fit indices for the proposed research model. ***Means 1% significance level.

**TABLE 7:** Results of structural equation modeling.

Hypothesis	Paths	β-coefficient	*t-*value
1	Environmental awareness → Environmental CSR content	0.180***	1.748
2	Social awareness → Environmental CSR content	0.174***	1.674
3	Influencer impact → Environmental CSR content	0.212	2.353
4	information sharing → Environmental CSR content	0.118**	1.087
5	Environmental awareness → Advertisement related content	0.326***	3.341
6	Social awareness → Advertisement related content	0.227**	2.159
7	Influencer impact → Advertisement related content	0.129**	1.141
8	Information sharing → Advertisement related content	0.285**	2.670
9	Environmental CSR content → Attitude to share content	0.302***	3.155
10	Advertisement related content → Attitude to share content	0.184***	1.941

**, *** means 5% and 1% significance level.

### Goodness of Fit Index

Because PLS-SEM does not produce a Goodness of Fit (GoF) value by default, the R2 value is frequently regarded as the primary source for evaluating a suggested structural model’s most sought-after explanatory capacity (Wang and Zhang, 2020; Janani et al., 2022). A contemporary diagnostic method, GoF = (AVE–R2), developed by Tenenhaus et al. (2005), has been used in recent studies to compute the Goodness of Fit (GoF) index in PLS-SEM. Following Tenenhaus et al. (2005), this study used the same method to calculate the Goodness of Fit (GoF) index, shown in Table 8. Goodness of Fit (GoF) values over 0.1, 0.25, and 0.36, according to Amorelli and García-Sánchez (2021), imply GoF small; GoF medium; and GoFlarge accordingly. Goodness-of-Fit (GoF) score of 0.624 indicates that our suggested structural model is well-fitted to the GoF large data set.

**TABLE 8:** Calculation of Goodness of Fit (GoF) index.

Latent construct(s)	AVE	*R* ^2^
Impact of influencers	0.514	
Social awareness	0.545	0.708
Environmental Awareness	0.561	0.751
Information Sharing	0.503	0.727
Attitudes	0.633	0.643
Average Scores	0.551	0.707
AVE × R^2^	0.390	
GoF = √(AVE × *R*^2^)	0.624	

*GoFsmall = 0.1; GoFmedium = 0.25; GoFlarge = 0.36.*

RETRACTED

## Conclusion and Policy Implications

Consumers’ online reviews from December last year were analyzed to see how the hospitality industry’s focus on CSR changed throughout that period. Although governments, businesses, and other stakeholders are interested in sustainability and CSR, customers don’t seem to share their enthusiasm. In addition, the results of this study show how the mood and rating of customer reviews are linked to CSR aspects. When people are exposed to environmental components, they tend to have more favorable feelings and higher scores in their reviews.

The findings of this study have substantial implications for both theory and practice. When customers interact with CSR material via social media, they are far more likely to associate themselves with a brand. This study gives actual evidence of this. People who use social media to receive and engage with CSR information are more likely to identify themselves as customers because they feel belonging and connected through social media (Basile and Vona, 2021). With this discovery, we better grasp social media’s function in establishing social identity than we did before.

A new mode of communication was used to investigate eWOM intention about CSR for the first time (i.e., social media). Consumer behavior and social media are better-understood thanks to a new mechanism that explains how CSR-related actions on social media lead to good eWOM intentions (Khan et al., 2021). As more businesses realize the value of social media marketing, it will grow in popularity (Elshabasy, 2018). This study contributes to the literature by confirming the relationship between consumers’ CSR-related social media behaviors and eWOM intentions.

### Policy Implications

#### Implications for Theory

Finding the variables that explain eWOM (intention to share and comment on CSR information) is the primary objective of this work. Studies on social and environmental consciousness have either focused on one or the other variable to explain pro-environmental or socially responsible behavior (Andersen and Skjoett-Larsen, 2009; Ge and Liu, 2015; Úbeda-García et al., 2021), or they have integrated social and environmental issues into only one construct. To better understand their position in the intention model, the current study looks at both values individually. Although prior studies have shown that social and environmental awareness are linked, empirical evidence shows that this is not the case (Quarshie et al., 2016).

It has been suggested that social and environmental consciousness can positively impact CSR communication since prosocial persons are more likely to analyze information and evaluate the message to a larger extent, employing central routes of evaluation. However, it’s possible to extend this theoretical reasoning to include negative publicity and well-intentioned but uncontrolled communication. Social networks can reward socially responsible enterprises by promoting them through CSR information (Yusliza et al., 2019).

RETRACTED

Our research adds to the body of knowledge on hospitality by proposing that the impact of eWOM is influenced by both the information and the individual. The general communication and marketing literature tends to analyze independent correlations between the proposed variables, therefore there is very limited empirical evidence about communication concerns related to CSR and even less in the hospitality sector. This study expands this line of research. Our findings show that eWOM intentions to comment and share on CSR news are positively influenced by information value, and self-disclosure.

Another finding that confirms previous research is that the quality of the content supplied affects people’s eWOM intentions (Serra-Cantallops and Salbi, 2014; Lee et al., 2015). The results of this study also highlight the importance of trust in fostering online conversation. In this study, trust was proven to be a critical factor in Wechat and social network users’ opinion-giving and opinion-passing behaviors regarding CSR issues. A previous study (Cheung, 2015; Gruzd Hernández-García, 2018) has shown that trust is a precondition for self-disclosure, as well as to increase the intention to comment on and share CSR posts, because it reduces (or even completely eliminates) the perceived risks involved in this interpersonal exchange situation.

#### Managerial Implications

1. According to this research, managers have three options for implementing change: There are two reasons for this: First, customers tend to find negative evaluations more informative than positive ones (Mattera et al., 2021; Yumei et al., 2021).
2. Second, firms should make their CSR commitments public so that others can learn about them. Customer reviews with CSR content could be used in CSR communication plans as a potential activity.
3. Companies should also begin actively involving customers in the creation of CSR value. Value co-creation begins with a user’s experience with the platform (Banks et al., 2014).
4. As previously mentioned, it’s also worth mentioning that pro-environmental conduct is more widespread in everyday activities. Because of this, the introduction of new government policies should create awareness and encourage customers to modify their behavior.
5. Consumer expectations can be assessed and incorporated into future CSR strategies by corporations. To avoid skepticism, organizations should verify that their CSR issues are presented and communicated truthfully before using public relations methods.
6. Organizations that are serious about promoting sustainability and corporate social responsibility (CSR) should cultivate their media relations and publish press releases on a regular basis to highlight the importance of their CSR and gain publicity.

RETRACTED

#### Limitations and Future Research

The study’s reliance on hypothetical consequences and self-reporting analyses is also a methodological drawback. In the future, it would be fascinating to investigate the study’s research goal in a real-world setting, even though the consequences-based survey has been employed in earlier studies in the hospitality context (e.g., lab experiments or field studies). To sum up, rather than examining actual behavior, this study focuses on participants’ intentions. Even though people’s actual behavior is influenced by their intentions (Stanislavská et al., 2020), it is recommended that future studies measure actual behavior. Only the variables of interest were examined in this study, and no other antecedents or consequences were considered.

## Data Availability Statement

The raw data supporting the conclusions of this article will be made available by the authors upon request.

## Author Contributions

All authors listed have made a substantial, direct, and intellectual contribution to the work, and approved it for publication.

## Conflict of Interest

The authors declare that the research was conducted in the absence of any commercial or financial relationships that could be construed as a potential conflict of interest.

## Publisher’s Note

All claims expressed in this article are solely those of the authors and do not necessarily represent those of their affiliated organizations, or those of the publisher, the editors and the reviewers. Any product that may be evaluated in this article, or claim that may be made by its manufacturer, is not guaranteed or endorsed by the publisher.

## Appendix

**TABLE A1:** Measurement scale.

Dimensions	Source	Constructs	Explanation
Impact of influencers	Ermeç, 2022	IMI 1 IMI 2 IMI 3	In my opinion, it has valuable information. In my opinion, it has a positive impression I think it is worth reading
Social awareness	Mar García-de los Salmones et al., 2021	SOAW 1 SOAW 2 SOAW 3	Posting personal experiences related to CSR activities on SNSs Posting or sharing photos, videos, memes, or gifs created by others related to CSR activities on SNSs. Posting or sharing photos, videos, memes, or gifs created by you related to CSR activities on SNSs.
Environmental Awareness	Mar García-de los Salmones et al., 2021	ENA 1 ENA 2 ENA 3 ENA 4	Customers are more concerned about environmental issues and relationships with suppliers. Environmental awareness moderates the link between CSR dimensions and positive e-WOM. From my point of view, environmental awareness positively influences consumers. In my opinion, it has interesting information
Information Sharing	Martínez et al., 2021	INSA 1 INSA 2 INSA 3 INSA 4	Posting from your SNS friends Comment on a friend’s social media post. Chatting with your SNS friends Like, share, or retweet from your SNS friends
Attitudes	Martínez et al., 2021	ATU 1 ATU 2 ATU 3	Online CSR communications are valuable and educational. Using the Internet for corporate social responsibility (CSR) messaging is beneficial. Online CSR communication helps in business development
